# Clinical Effect of Ear Endoscopic Intervention on CMEC Patients and Analysis of the Relationship between ROS, P-Akt, and HIF-1*α* Expression and the Degree of Bone Destruction

This article has been retracted.

**DOI:** 10.1155/2022/9931388

**Published:** 2022-09-10

**Authors:** Ming Yang, Longqiu Yang, Lang Wan, Qiuping Sun

**Affiliations:** ^1^E.N.T. Department, The First Hospital of Nanchang City, Nanchang 330006, China; ^2^E.N.T. Department, Huangshi Central Hospital, Affiliated Hospital of Hubei Polytechnic University, Edong Healthcare Group, Huangshi 435000, China

## Abstract

The clinical efficacy of ear endoscopic intervention in patients with congenital middle ear cholesteatoma (CMEC) is explored, and the relationship between the expression of reactive oxygen species (ROS), phosphorylated protein kinase B (P-Akt), hypoxia-inducible factor-1 *α* (HIF-1*α*) and the degree of bone damage are analyzed. A total of 72 CMEC patients admitted to the otolaryngology department of our hospital from 2019 to January 2021 for surgical treatment are selected. According to the different intervention methods, the microscope group and the otolaryngology intervention group are established, respectively, with 36 patients in each group. The patients in the microscope group are treated with a microscope for middle ear cholesteatoma surgery, and the patients in the otoscope intervention group are treated with an otoscope for middle ear cholesteatoma surgery. The experimental results show that ear endoscopic intervention has better clinical efficacy for CMEC patients, which can effectively shorten the operation time, reduce the incidence of postoperative complications, and effectively improve the hearing of patients.

## 1. Introduction

Congenital middle ear cholesteatoma (CMEC) is not common in clinical practice, but with the continuous improvement of technological level in the medical field and the improvement of the awareness and diagnosis level of otolaryngology on this disease, clinical reports of CMEC cases are increasing, and the surgical treatment methods for this disease are constantly optimized and improved [1, 2]. Before the clinical use of microscope surgical intervention treatment, due to the particularity of middle ear cholesteatoma disease location, microscope interference technique is likely to cause damage to the ear bone in the process and the gas room is bigger; the physiological structures of the middle ear and external ear parts of patients are relatively complex, and simple application of the microscope with surgical treatment is likely to destroy the normal tissue structures of the ear. It is also possible that intraoperative cholesteatoma may not be completely removed, and cholesteatoma may easily remain in hidden sites such as the anterior and facial crypts of the superior tympanic cavity and tympanic sinus [3, 4].

Otoendoscopic intervention is an important product of the continuous improvement of otorhinolaryngology treatment technology in the medical field in recent years, showing certain advantages in the treatment of middle ear lesions, but there are few studies related to the clinical efficacy of this operation on CMEC [5]. Based on this, this study aims to explore the clinical efficacy and safety of otoscopy intervention for CMEC patients, and explore the relationship between reactive oxygen species (ROS), phosphorylated protein kinase B (P-Akt), hypoxia-inducible factor-1*α* (HIF-1*α*) expression, and the degree of bone damage based on the recurrence mechanism of patients, aiming to provide an effective basis for clinical optimization and improvement of diagnosis and treatment model.

The rest of this paper is organized as follows: Section 2 discusses related work, followed by the surgical methods and detection methods designed in Section 3.  Section 4 shows the experimental results and analysis, and Section 5 gives the conclusion of this study and puts forward the direction of the follow-up research.

## 2. Related Work

With the continuous improvement of technology in the medical field, the diversification of treatment techniques for middle ear cholesteatoma has been effectively promoted, but the efficacy and prognosis of different surgical methods for patients are also different [6]. In the past, clinicians mostly used microscopes for interventional therapy, which to some extent improved the success rate of surgery, improved the effectiveness of surgery, and ensured targeted adjuvant therapy for patients after surgery to improve clinical efficacy [7]. It should be noted that although microscopic surgery can achieve a certain therapeutic effect, the improvement of patients' hearing is slow and postoperative recurrence is easy to occur, which hinders the recovery of patients [8]. From the perspective of biological histology, the accumulation of highly proliferative squamous epithelium is the main pathological feature of CMEC patients. With the continuous increase of cholesteatoma, negative pressure and bag-like entrapment of the tympanum can be caused, and a hypoxia microenvironment can be formed. Hif-1 *α* is a functional unit of hypoxia-inducible factor-1, which can increase the expression products of these genes by regulating hypoxia-response-related genes and thus exert relevant biological effects [9].

In recent years, there are many studies on hiF-1 *α* in neoplastic diseases, but there are few studies on hiF-1 *α* in middle ear cholesteatoma. ROS is distributed in various tissues and cells. These studies have found that when the body suffers from hypoxia or inflammatory stimulation, the mitochondria of cells can produce excessive ROS, which will bring a series of changes to the biological functions of the body cells and tissues [10]. It suggests that the above indicators have a certain impact on the occurrence and development of CMEC, but there are still few relevant studies at present, and the mechanism of the occurrence and development of CMEC is also one of the main topics of clinical research.

Ear endoscopic surgery is a new type of surgical treatment, mainly through ear endoscopy-assisted observation of patients' lesions, in order to reduce the damage of the patient's lesions, and then achieve the purpose of treatment. Compared with microscopic surgery, ear endoscopy can better expand the surgical field of vision, reduce the damage to patients, shorten the length of hospital stay, and find the parts that cannot be seen under the microscope, which is more minimally invasive and easier to be accepted by patients [11]. The results of this study are similar to those of previous studies. Compared with the microscope method, the intervention of otoscopy can effectively shorten the operation time, reduce the risk of postoperative complications, and have a more obvious hearing recovery effect. Therefore, we can summarize the advantages of otoendoscopic surgery as follows: otoendoscopic intervention uses an external auditory canal approach to effectively reduce the damage to normal tissue structure and promote rapid postoperative recovery of patients. Due to the small diameter of the ear endoscope, after entering through the normal passage of the external auditory canal, physicians can better adjust the angle of the ear endoscope to observe the surgical field, which can fully expose the specific structure of the middle ear, especially the middle ear crypt, and greatly reduce the surgical residue.

In addition, this study focused on the occurrence and development mechanism of middle ear cholesteatoma, and combined with the analysis of previous clinical literature, suggesting that it may be formed in an obvious hypoxia environment. The results of this study showed that ROS and P-Akt expressions were higher in cholesteatoma than in normal skin, which suggested that ROS mainly played a role in promoting cell proliferation during the formation of middle ear cholesteatoma. In this study, HIF-1*α* expression was detected in the epithelium of middle ear cholesteatoma and skin of the external auditory canal, and it was observed that the expression of HIF-1*α* in cholesteatoma was significantly higher than that in the skin of external auditory canal. Previous studies have reported that chronic inflammation of the mastoid air chamber can lead to mucosal hypertrophy and accumulation of sticky secretions, which affects middle ear ventilation and drainage and leads to hypoxia in middle ear tissues [12, 13]. The results of this study suggest that hypoxia in cholesteatoma can activate HIF-1*α* expression. In addition, Spearman correlation analysis showed that the degree of bone destruction in cholesteatoma was positively correlated with the expression of ROS-Akt and HIF-1*α*, which suggested that the degree of bone destruction in cholesteatoma was closely related to the expression of the above three indicators. It is suggested that the above three indicators can be used for the corresponding detection to evaluate the disease development of patients, which is of great significance for the subsequent development and improvement of effective diagnosis and treatment plans.

## 3. Surgical Methods and Detection Methods

A total of 72 CMEC patients admitted to the otolaryngology department of our hospital from January 2019 to January 2021 for surgical treatment are selected. According to different surgical intervention methods, the microscope group and the otoscopy intervention group are established, respectively, with 36 patients in each group. There are 16 males and 20 females in the microscope group, aged from 12 to 40 years, including 4 children, with an average age of (23.15 ± 2.83) years. All patients in the microscope group have unilateral disease. In the ear endoscopy intervention group, there are 17 males and 19 females, aged from 11 to 38 years, including 3 children, with an average age of (22.84 ± 3.03) years. All patients in the group have unilateral disease. There are no significant statistical differences in baseline data of the two groups, including gender, age, and nature of the disease (all *P* > 0.05), which confirmed that the comparison between groups is scientific and reasonable.

The patient inclusion criteria are as follows: (1) all patients included in this study meet the diagnostic criteria for middle ear cholesteatoma [14]; (2) clinical imaging diagnosis shows that the patient's tympanic membrane is intact without any signs of tympanic membrane perforation; (3) the patients have no history of otorrhea or middle ear surgery; (4) all have progressive hearing loss.

The patient exclusion criteria are as follows: (1) eustachian tube mouth closed; (2) patients with facial paralysis; (3) the deaf; (4) poor clinical compliance or withdrawal from the study due to various reasons.

### 3.1. Surgical Methods

The patients in the microscope group are treated with a microscope for middle ear cholesteatoma surgery, and the specific steps are as follows: group patients receive general anesthesia, after tracheal intubation and take the patient supine, regular disinfection draping is performed, after the operating room had been used for patients, a puncture of 0.5cm is made on the ear parallel to the ditch after ear arc incision, a square flap muscle is cut and subcutaneous tissue is left to spare, making the mastoid left fully exposed outside, up to the line, next to the mastoid tip. After that,, the mastoid cortex is fully excised to the body surface projection of the sigmoid sinus, and the mastoid cavity, tympanic sinus, and epitympanic chamber are opened successively, and all lesions in the tympanic sinus, mastoid cavity, and tympanic chamber are completely removed. The ossicular chain is examined with a microscope and reconstructed with the corresponding treatment. The eardrum is repaired with epistomatous fascia and fixed with a gelatin sponge. The patients in the ear endoscopy intervention group are treated with ear endoscopy for middle ear cholesteatoma surgery, and the specific steps are as follows: the patients under general anesthesia and general anesthesia patients supine, head to the contralateral, lateral plane, auricle surrounding mucosa iodine disinfection three times, draping, along the external auditory canal under endoscope cartilage and ear cavity gap into the needle, an external auditory canal subcutaneous local infiltration anesthesia, along the skin and mucous membrane under endoscope border do before after the arc incision, external auditory canal bone exposure, peel the mucous membrane to expose the drum ring, lift the bone ring to expose the tympanum, chisel out the posterior superior wall of the external auditory canal, expose the superior tympanum, open the tympanum sinus and the mastoid cavity along the superior tympanum, remove the lesions in the superior tympanum sinus and the mastoid cavity, explore the ossicular chain and reconstruct the ossicular chain, repair the tympanum with the musculofascial. For reduction of the mucous membrane, if more bone is removed, the mucous membrane can be affixed to the sinus tympanum and mastoid cavity, and an iodoform gauze strip is used to fill the surgical cavity. All patients received an intravenous infusion of antibiotics after surgery, and iodoform gauze strips are removed from the external auditory canal 3 weeks after surgery. All patients are followed-up for 6 months.

### 3.2. Detection Methods

With the informed consent of all patients, 68 cholesteatoma specimens are collected intraoperatively, and the mild group (*n* = 36) and severe group (*n* = 32) are established according to the degree of bone damage. Meanwhile, 30 cases of normal external auditory canal bone tissue are randomly selected as the control group.

#### 3.2.1. ROS Expression Detection Method

The samples and normal skin tissues are frozen, sliced, and rewarmed. All samples are dried and fixed with paraformaldehyde for 10 min. After the paraformaldehyde is completely dried, they are washed by shaking on a decolorizing shaker 3 times in PBS (pH7.4), 5 min for each time. The tissue sections are placed in the repair box filled with EDTA antigen repair buffer PBS (pH8.0) for antigen repair in a microwave oven for 10 min with low heat. After natural cooling, the slides are placed in PBS (pH7.4) and washed by shaking on a decolorizing shaker 3 times, 5 min each. After the sections are slightly shaken dry, a histochemical pen is used to draw circles around the tissues. PBS is shaken dry, and BSA is dropped and sealed for 30 min. The sections are stained with ROS fluorescent probe-dihydroxyethylene. The sections are placed flat in a wet box and incubated at 4°C overnight. The slides are placed in PBS (pH7.4) and washed by shaking on a decolorizing shaker 3 times, 5 min each. The slices are briefly shaken dry and sealed with antifluorescence quenching sealing tablets. The sections are observed under a fluorescence microscope and the collected images (excitation wavelength of CY3 is 510∼560 nm, the emission wavelength is 590 nm, and red light is emitted) are analyzed semiquantitatively by image-pro Plus 6.0 Image analysis software. The interpretation of ROS frozen section immunofluorescence detection results is that after directly sealing the sheet, it shows red under the fluorescence microscope.

#### 3.2.2. P-Akt Protein Expression Detection Method

All obtained samples are extracted for protein extraction, a 100 mg tissue sample is placed in a 1–2 ml homogenizer, and the tissue is cut into pieces as far as possible with scissors (sterile). Add 400 *μ*L single detergent cracking solution (including PMSF) in a homogenizer, put on ice after the homogenizing operation, 5 minutes later the ice is crushed again, repeat this process several times to ensure that the tissue is crushed to make the tissue as crushed as possible. After cracking for 30 min, the cracking liquid is transferred to a 2 mL centrifuge tube with a pipette and centrifuged at 12,000 rpm at 4°C for 5 min. The supernatant is divided into a 0.5 ml centrifuge tube and stored at −20°C for inspection. According to the molecular weight of the target protein, 10% SDS-PAGE gel is prepared for vertical electrophoresis, and the loading amount is adjusted according to the protein concentration, keeping 45 *μ*g protein loading per well. The sample protein is concentrated at a voltage of 90 V for 1 h and then separated by electrophoresis at a voltage of 120 V and 100 min. After electrophoresis, the PVDF membrane is immersed in pure methanol for 10 min and deionized water for 20 min and transferred to the PVDF membrane at a constant pressure of 100 V for 120 min. The shaker is closed with 5% skim milk powder for 1.5 h at room temperature, and the membrane is washed with PBS liquid 3 times, 15 min each time. Then, P-Akt and internal reference GAPDH antibodies are diluted strictly according to the instructions and incubated at 4°C overnight. The film is washed with TBST solution 3 times, 15 min/time, and the secondary antibody is added, and the bed is shaken at room temperature for 2 h. The ECL color solution is used for color development and fixer solution is used to terminate color development. Each experiment is repeated 3 times.

#### 3.2.3. HIF-1*α* Expression Detection Method

Application of the above to obtain tissue samples of patients and complete fixed with 10% formalin fixation fluid, using paraffin embedding and serial section, after drying, after the slice for regular dewaxing process, hydration, gradient ethanol distilled water rinse after soaking in the PBS, 3% hydrogen peroxide deionized water incubation, high-pressure antigen repair, goat serum incubated with the working fluid. After incubation at room temperature, PBS is washed, and horseradish enzyme-labeled streptomycin ovalbumin working solution is added. After incubation at room temperature, PBS is cleaned, DAB is developed, hematoxylin is restained after rinsing with distilled water, and xylene is transparent and sealed. The expression of HIF-1*α* in cholesteatoma and normal tissues is detected. Positive cell count is performed in 5 fields under 400x magnification, and the proportion of positive cells is calculated. Criteria: (−): <10% (+): the number of positive cells is 10%–25% (++): the number of positive cells is 26%–50% (+++): positive cell number >50%.

### 3.3. Observation Indicators

Intraoperative and postoperative indicators are compared between the two groups, including operation time, postoperative complications, and surgical success rate. The hearing changes of the two groups are compared before and 6 months after surgery. The expression of ROS, P-Akt, and HIF-1*α* in each group is compared. The correlation between ROS, P-Akt, HIF-1*α* expression, and the degree of bone destruction in CMEC patients is analyzed.

### 3.4. Statistical Methods

SPSS 26.0 software is used to complete effective processing of the data in the study. The measurement data are tested for normality and homogeneity of variance to meet normal distribution. The mean ± standard deviation ($\bar{x}$ ± *s*) is used to represent the data, and the *t*-test is performed. Spearman correlation coefficient is used to analyze the correlation between the expression of ROS, P-Akt and HIF-1*α*, and the degree of bone damage in CMEC patients. *P* < 0.05 indicates the statistical difference in data comparison.

## 4. Experimental Results and Analysis

### 4.1. Comparison of Intraoperative Indicators and Postoperative Complications

Table 1 shows the comparison of intraoperative indicators and postoperative complications. It can be seen from Table 1 that compared with the microscope group, the operation time of CMEC patients receiving otoscopy intervention is significantly shorter, the incidence of postoperative complications decreases significantly than in the microscope group, and the success rate of surgery increases significantly (all *P* < 0.05).

### 4.2. Comparison of Hearing Changes before and 6 Months after Surgery

Table 2 shows the comparison of hearing changes. In Table 2, ^*∗*^ represents a comparison with before surgery, *P* < 0.05. It can be observed from Table 2 that there are no statistically significant differences before surgery (*P* > 0.05), and the index values decrease significantly 6 months after surgery. The inter-group comparison shows that the index values of the otoscopy intervention group decrease significantly than the microscope group (all *P* < 0.05).

### 4.3. Comparison of the Expression of ROS, P-Akt, and HIF-1*α*

Table 3 shows the ROS, P-Akt, and HIF-1*α* expressions in each group.  Table 4 shows the comparison of HIF-1*α* expression in each group. Through the above experimental results, it can be observed that the levels of ROS, P-Akt, and HIF-1*α* in severe and mild groups are significantly higher than those in the control group, and those in the severe group decrease significantly than those in the mild group (*P* < 0.05). The percentage of HIF-1*α* expression in cholesteatoma cells is (++) and (+++), which indicates that the severe group and mild group increased significantly, and the severe group significantly increases than the mild group (*P* < 0.05).

### 4.4. Correlation between ROS, P-Akt, and HIF-1*α* Expression and the Degree of Bone Damage in Patients

Table 5 shows the correlation between ROS, P-Akt, HIF-1*α* expression, and the degree of bone damage. It can be seen from Table 5 that the Spearman correlation coefficient is used to analyze the correlation between the degree of bone destruction and the expression of ROS, P-Akt, and HIF-1*α* in patients, which shows a positive correlation (*P* < 0.05).

## 5. Conclusion and Future Work

The clinical efficacy of ear endoscopic intervention in patients with CMEC is explored, and the relationship between the expression of ROS, P-Akt, HIF-1*α*, and the degree of bone damage is analyzed. Ear endoscopic intervention has better clinical efficacy for CMEC patients and is worthy of clinical application. At the same time, this study conducts an in-depth research on the occurrence and development mechanism of middle ear cholesteatoma disease, confirming that the degree of bone destruction is significantly correlated with ROS, P-Akt, and HIF-1*α*, and suggests that hypoxia can promote the proliferation of cholesteatoma cells. The disease progression and disease of such patients can be determined by detecting the above indicators. It can also develop and improve the diagnosis and treatment plan around it, and then improve the clinical efficacy of patients. The study provides a new target and idea for the prevention and treatment of cholesteatoma.

## Figures and Tables

**Table 1:** Comparison of intraoperative indicators and postoperative complications.

Group	The operation time (min)	Postoperative complications (*n*, %)	Surgical success rate (*n*, %)
Microscope group (*n* = 36)	72.16 ± 10.72	10 (27.78)	25 (69.44)

Ear endoscopy intervention group (*n* = 36)	55.69 ± 9.16	2 (5.56)	33 (91.67)

*t/x* ^2^	7.008	6.400	5.675

*P*	＜0.001	0.011	0.017

**Table 2:** Comparison of hearing changes.

Group	Bones poor guide (dbHL)		Air guide valve level (dbHL)	
	Before the operation	6 months after surgery	Before the operation	6 months after surgery
Microscope group (*n* = 36)	32.47 ± 6.25	21.64 ± 3.72^*∗*^	49.86 ± 6.25	36.41 ± 5.12^*∗*^
Ear endoscopy intervention group (*n* = 36)	33.04 ± 6.83	13.62 ± 3.18^*∗*^	50.25 ± 6.93	24.18 ± 4.76^*∗*^
*T*	−0.369	9.833	−0.251	10.497
*P*	0.713	＜0.001	0.803	＜0.001

**Table 3:** ROS, P-Akt, and HIF-1*α* expressions in each group.

Group	ROS fluorescence expression value	P-Akt expression
Severe group (*n* = 36)	101.52 ± 15.64	0.93 ± 0.08
Mild group (*n* = 32)	78.64 ± 11.83	0.71 ± 0.06
The control group (*n* = 30)	47.38 ± 6.94	0.52 ± 0.04
*F*	9.413	7.883
*P*	＜0.001	＜0.001

**Table 4:** Comparison of HIF-1*α* expression in each group.

Group	(−)	(+)	(++)	(+++)
Severe group (*n* = 36)	17.03 ± 3.01	28.18 ± 3.51	35.47 ± 4.02	30.18 ± 3.62

Mild group (*n* = 32)	25.45 ± 3.22	26.26 ± 3.24	23.71 ± 3.68	26.04 ± 3.29

The control group (*n* = 30)	52.17 ± 6.28	21.84 ± 2.93	16.76 ± 2.46	12.17 ± 2.04

*F*	−12.251	5.870	9.478	11.092

*P*	＜0.001	＜0.001	＜0.001	＜0.001

**Table 5:** Correlation between ROS, P-Akt, and HIF-1*α* expression and the degree of bone damage.

	Degree of bone destruction	
	rs	*P*
ROS	0.754	＜0.001
P-AKT	0.739	＜0.001
HIF-1*α*	0.802	＜0.001

## Data Availability

The simulation experiment data used to support the findings of this study are available from the corresponding author upon request.
